# *CircNF1-419* improves the gut microbiome structure and function in AD-like mice

**DOI:** 10.18632/aging.102614

**Published:** 2020-01-06

**Authors:** Chen Diling, Qi Longkai, Guo Yinrui, Liu Yadi, Tang Xiaocui, Zhu Xiangxiang, Zeng Miao, Li Ran, Shuai Ou, Wang Dongdong, Xie Yizhen, Yuan Xujiang, Burton B. Yang, Wu Qingping

**Affiliations:** 1 State Key Laboratory of Applied Microbiology Southern China, Guangdong Provincial Key Laboratory of Microbial Culture Collection and Application, Guangdong Open Laboratory of Applied Microbiology, Guangdong Institute of Microbiology, Guangdong Academy of Sciences, Guangzhou 510070, China; 2 Guangdong Pharmaceutical University, Guangzhou 510006, China; 3 Guangxi University of Chinese Medicine, Nanning 530023, China; 4 Academy of Life Sciences, Jinan University, Guangdong Province, Guangzhou 510000, China; 5 Chengdu University of Traditional Chinese Medicine, Chengdu 610075, China; 6 Department of Physiology, Shantou University Medical College, Shantou 515063, China

**Keywords:** circular RNAs, microbiome-gut-brain axis, dietary interventions, gut microbiome, therapeutic markers

## Abstract

Our pre-experiments found that the brain circRNA sequence profiles and gut microbiota in AD-like mice were changed, as circNF1-419 could enhance autophagy to ameliorate senile dementia in AD-like mice, so we conclude that there might some connections between circRNA and gut microbiome. Therefore, we use the over-expressed *circNF1-419* adeno-associated virus (AAV) animal system with the aim of identifying possible connections. Our results showed that over-expression of circ*NF1-419* in brain not only influenced the cholinergic system of brain, but also changed the gut microbiota composition as the *Candidatus Arthromitus*, *Lachnospiraceae FCS020 group*, *Lachnospiraceae UCG-006*, and [Eubacterium] *xylanophilum group*, and the intestinal homeostasis and physiology, and even the gut microbiota trajectory in new born mice. These findings demonstrate a link between circRNA and gut microbiome, enlarge the ‘microbiome- transcriptome’ linkage library and provide more information on gut-brain axis.

## INTRODUCTION

The microbiota-gut-brain axis integrates neural, hormonal and immunological signaling between the gut and brain, and has a profound effect on mammalian growth and health throughout life [1, 2]. However, systematic linkage of the two distant organs and the physiological and pathological impacts of the microbiota-gut-brain axis on growth and health remain largely unclear. Extensive research is required to validate existing routes of bidirectional communication, to identify new connections, and to illuminate the relevant molecular mechanisms. In previous studies, we found that alterations of gut microbiota and transcriptomes of the small intestine and brain are accompanied by changes in the concentrations of Aβ_1-42_ in the hippocampal CA1 region [3]. Furthermore, probiotics of fructo-oligosaccharides from natural herbs could modulate these interactions between gut ecology and brain physiology [3], indicating that the gut microbiota and brain interact with each other. However, additional evidence is needed, particularly clinical sample support, and the mechanism remains poorly understood and requires further investigation.

Research increasingly suggests that diet and lifestyle are important factors for human health. A vast array of paradigms have confirmed that many common diseases are more or less related to obesity, such as sleep apnea [4], infertility [5], diabetes [6], hypertension [7], coronary heart disease [8], liver disease [9, 10], osteoporosis [11], cancers [12, 13], and even Alzheimer’s disease (AD) [14]. Weight management is therefore particularly important for keeping healthy. In traditional concepts, body weight (or more accurately, body fat) is considered to be regulated by the central nervous system (CNS). However, recent studies have confirmed that symbiotic microorganisms also play an important role regarding fluctuations in energy status [15–18], and fecal microbiota transplantation could influence acute feeding behavior and long-term energy homeostasis [19, 20]. Within this symbiotic interaction, a clear understanding of who drives decisions about when, how much, what and why is lacking.

Circular RNA (circRNA) is a type of single-stranded RNA which, unlike the better known linear RNA, forms a covalently closed continuous loop, i.e., in circular RNA the 3′ and 5′ ends normally present in an RNA molecule have been joined together [21]. This feature confers numerous properties to circRNAs, many of which have only recently been identified. As circRNAs do not have 5′ or 3′ ends, they are resistant to exonuclease- mediated degradation and are presumably more stable than most linear RNAs in cells. CircRNAs have been categorized as noncoding RNA, but more recently, they have been shown to encode proteins [22–24]. Like many other alternative noncoding isoforms, the biological functions of most circRNAs are unclear, however they have benefited from the development of high-throughput sequencing technology, which has enabled large-scale studies on circRNAs in recent years. Subsequent studies revealed that the expression of circRNAs is developmentally regulated, tissue- and cell-type specific, and shared across the eukaryotic tree of life [25–27]. CircRNAs are emerging as a heterogeneous class of molecules involved in modulating gene expression by regulating transcription and protein and miRNA functions. Studies have shown that in the brain, where the level of circRNA is significantly higher, some circRNAs consist mainly of portions of the multi-exon 5′ untranslated region (5′UTR), suggesting that functions of these multi-exon 5′UTR of genes and/or circRNA is new [28]. Increasing numbers of circRNAs function in the brain, including *circPDE4B* [29], *circRNA-0044073* [30], and *circHIPK3* [31], as well as in heart failure [32, 33], human cancer (Josh N, et al.) [34] and other diseases [35], suggesting that circRNAs are crucial functional molecules in mammals. Thus, studying the roles of circRNAs on the gut-brain axis is important. A forward chemical genetic screen revealed gut microbiota metabolites that modulate host physiology [36], and circRNAs were found to be degraded by RNase L when induced by poly(I:C) or infected by virus (Liu Y, et al.).

From these findings, we concluded that the gut microbiome may influence the expression of circRNAs, but experimental evidence for this is lacking. In our recent study, we showed that *circNF1-419* could regulate autophagy in over-expressing *circNF1-419* transfected astrocytes, likely through PI3K-I/Akt-AMPK-mTOR and PI3K-I/Akt-mTOR signaling pathways. And an AAV packaging system (virus titer 1 ×1 0^12^) over-expressing *circNF1-419* in vivo showed autophagy enhancing activity by binding Dynamin-1 and AP2B1, delaying senile dementia by regulating aging markers (p21, p35/25, p16) and inflammatory factors (IL-6, IL-10, NF-κB), and by reducing the expression of AD marker proteins Tau, p-Tau, Aβ_1-42_, and APOE in SAMP8 mice [37]. Therefore in this study, we subjected data on the gut microbiota and circRNA sequences of brain tissues from AD-like mice to choice-based conjoint analysis. In addition, from the preventive medicine perspective, considering the effects of diet on health and the causes and processes of chronic disease formation, we also focused on the influence of circRNAs in the brain to the gut and gut microbiome. We aimed to identify more associations between gut microbiota and brain circRNAs. We also aimed to enlarge the ‘microbiome-transcriptome’ linkage library, which would provide more information on the interplay between gut and brain in order to aid in the identification of potential therapeutic markers and mechanistic solutions to complex problems commonly encountered in pathology, toxicology, and drug development studies.

## RESULTS AND DISSCUSSION

### Gut microbiota plays an important role in the circRNA sequences in AD-like mice

To understand the network of circRNAs acting on the microbiome-gut-brain axis, the gut microbiota (Supplementary Figure 1A–1B), serum metabolites (Supplementary Figure 2A–2B), and circRNA sequences of brain tissues (Supplementary Table 1) from 8-month-old APP/PS1 mice were subjected to choice-based conjoint analysis. The interactions of gut microbiota and metabolites are shown in Figure 1A–1B, which revealed that *Adlercreutzia* (Actinobacteria), *Streptococcus*, *Lactobacillus,* *Ruminococcus* and *Prevotella* may be the key bacteria regulating serum metabolites such as L-acetylcarnitine, 11-beta-hydroxyandrosterone- 3-glucuronide, phosphatidylethanolamine and phosphorus esters. With the gut microbiota and serum metabolite changes, there were 501 differentially expressed circRNAs in the model group (fold change > 1.50, *p* < 0.05 vs normal C57 mice, Figure 2A) up-regulated, and 624 circRNAs down-regulated, including chr14_84532875_ 84533695_+ (*Pcdh17*), chr1_140425193_ 140450304_+ (*Kcnt2*), chr8_94047272_ 94055344_+ (*Ogfod1*), chr3_158104428_ 158148699_- (*Lrrc7*), chr10_62633977_ 62643372_- (*Ddx50*), chr12_69603476_69607412_- (*Sos2*), chr12_85028770_85030887_+ (*Ylpm1*), chr10_93208172_93218089_+ (*Cdk17*), chr11_79546971_79551134_+ (*NF1*), and chr6_52609145_52630349_- (*Hibadh*); more details are shown in Supplementary Table 1, (PRJNA553830).

**Figure 1:** **The combined data analysis between gut microbiome and serum metabolome of APP/PS1 mice.** (**A**) The Spearman correlation coefficient for each metabolite type and each bacterial genus, see also Supplementary Figure 1A–1B and Supplementary Figure 2A–2B. (**B**) Serum metabolome and genera. Red and blue indicate positive and negative correlations, see also Supplementary Figure 1A–1B and Supplementary Figure 2A–2B. Hub nodes with the most connections are highlighted in red. Data are presented as the means of more than 6 independent experiments.

**Figure 2:** (**A**) Differentially expressed circRNAs in the APP/PS1 double transgenic mice brain samples (fold change > 1.50, p < 0.05 vs normal C57 mice, n=3). (**B**) Differentially expressed mRNAs in the APP/PS1 double transgenic mice brain samples (fold change > 1.50, p < 0.05 vs normal C57 mice, n=3). (**C**) Rarefaction curves based on OTU. The structure at the (**D**) phylum and (**E**) genus levels. (**F**) Histopathological changes in the brain identified using H&E staining and biomarker expression of Tau and Aβ_1-42_ using immunohistochemical methods after fecal microbiota from six months APP/PS1 mice transplantated into 9 months old C57 mice, (n≥6).

Given that the function of most circRNAs is unknown, the mRNA sequence was concurrently analyzed to offer an alternative explanation. Using RNA-sequencing, 347 genes were up-regulated and 507 genes were down-regulated (fold change > 1.50, *p* < 0.05, Figure 2B) in brain tissues dissected from APP/PS1 double transgenic mice. The networks of Ingenuity Canonical Pathways (IPA) data showed that the diseases and functions of cellular movement, cell death and survival might be regulated by molecules in a network including 26s Proteasome, *AGT*, *ALB*, *BCR* (complex), *BLNK*, *CA3*, *CASP1*, *CCND2*, *CD4*, *CDT1*, *CENPF*, *DAPK1*, *DIO2*, *DSP*, *EGR1*, Focal adhesion kinase, *FST*, *HGF*, *IgG*, *KDELR3*, *KIF22*, *LBX1*, *LY9*, *MAPK12*, *MMP19*, *NEU4*, *NOD2*, *P38* and *MAPK*, *PRNP*, *RIN1*, *S100A8*, *S100A9*, *SDC1* and *ST14*; cell-to-cell signaling and interaction, nervous system development and function, cellular function and maintenance might be regulated by molecules in a network including *Akt*, *Alp*, *CAMK2A*, *CAMK2N1*, *CCKBR*, *CHRM3*, *CLEC7A*, *CSF2RB*, *CYBB*, *EPHA4*, *ERK*, *FGF7*, *FLT3*, *FOSL2*, *Growth hormone*, *IL23*, *IRX1*, *KCNA5*, *KLF10*, *MAPK*, *MGLL*, *MIA*, *MMD*, *NPY*, *PLK2*, *PPP1R1B*, *RAG1*, *RGS4*, *RORC*, *SNCA*, *SPARC*, *STAT5a/b*, *TLR2*, *VEGF*, *WNT9A* mRNAs (Supplementary Figure 3). Additional studies are needed in this area.

GO (gene ontology) enrichment analysis of differentially expressed circRNAs showed that they mainly influenced synaptic transmission, post-synapse, positive regulation of neurogenesis, single-organism behavior, protein serine/threonine kinase activity, histone modification, regulation of GTPase activity, and neuron death. KEGG enrichment analysis showed that they mainly influenced *MAPK*, *Rap1*, *cAMP*, glutamatergic synapse, neurotrophin and Rap1 signaling pathways. Reactome enrichment analysis of differentially expressed circRNAs showed that they mainly influenced developmental biology, signaling by Rho GTPases, neuronal system, signaling by NGF, axon guidance, signaling by EGFR, transmission across chemical synapses, NGF signaling via TRKA from the plasma membrane, organelle biogenesis and maintenance, and signaling by FGFR1~4. Bioinformatics analyses of circRNA and mRNA annotation, functional classification, functional enrichment and cluster analyses showed that the changes of gut microbiota and serum metabolites could influence the circRNA sequences and function. This conclusion requires additional evidence, particularly clinical sample support, and the mechanism remains poorly understood and needs further investigation.

In order to understand the connections between the gut microbiota and brain function, an additional experiment was carried out using fecal microbiota transplantation. Fecal samples were collected from 8-month-old APP/PS1 mice, PBS was added and the bacterial solution was concentrated immediately by centrifugation. C57 mice (9 months old) were treated with the bacterial solution by enema, for 3 weeks, after the mixture of antibiotics according to the method of de Groot PF, et al. [59]. Microbiome analysis of the 16S rRNA genes was performed after 3 months. Gut microbiota from the APP/PS1 mice settled in the normal mice (Figure 2C–2E), influenced the intestinal microenvironment (Figure 2F, H&E of intestine), and up-regulated the expression of Tau and Aβ_1-42_ (Figure 2F) in the hippocampus. Together these results and those of our previous study demonstrating that the most highly abundant gut microbiota were correlated with the level of Aβ_1-42_ [3], led us to summarize that the gut microbiota have some interactions with the circRNA sequences of the brain in AD-like mice, and targeting the gut microbiota might be a feasible and effective strategy for ameliorating the symptoms or even delaying the progression of AD. Thus the gut microbiota plays an important role in the progression of AD.

### *CircNF1-419* changes the intestinal physiology and gut microbiota in SAMP8 mice

Recently, a report demonstrated that avian leucosis virus targets circ-Vav3 and then sponges gga-miR-375 to promote epithelial-mesenchymal transition [38], indicating that a microorganism could directly influence the formation, expression and function of circRNAs, and the mysterious of circRNA is suggested in increasing numbers of studies [30, 38, 39]. In order to verify these, the expression level of circRNAs was examined by qRT-PCR in AD-like mice (PCR primers are listed in Table 1). The circRNAs of *circ_zfyve1-504*, *circ_zcchc11-811*, *circ_zfp652-1147*, *circ_zfp236-1257*, *circNF1-419* and *circ_zranb1-1575* were differentially expressed (Figure 3A), suggesting that these circRNAs may be related to AD. We then over-expressed *circNF1-419* and *circ_0001239* in the animal brain using an adeno-associated virus (AAV) system, with the aim of identifying possible connections.

**Table 1:** PCR primers.

**Primer name**	**Sequence (5′->3′)**	**Product size (bp)**
β-actin	β-actin-F1: GCTTCTAGGCGGACTGTTAC β-actin-R1: CCATGCCAATGTTGTCTCTT	100
Circ-Zfyve1	Circ-Zfyve1-F1: 5′- tcagcttctgggttctggtaaca-3′ Circ-Zfyve1-R1: 5′- gtgtgtgagactttccatcacc-3′	123
Circ-Zranb1	Circ-Zranb1-F2: 5′- gttattaagcacaagatctgc-3′ Circ-Zranb1-R2: 5′- gctgcttgctgagataccttt-3′	135
Circ-Zcchc11	Circ-Zcchc11-F1: 5′- cagcagatgatttgatttgc-3′ Circ-Zcchc11-R1: 5′- atattcttctttggttcatg-3′	159
Circ-Zfp652	Circ-Zfp652-F1: 5′- agcacatgaacgttactcac-3′ Circ-Zfp652-R1: 5′- cttggagcatcttgtctgaatg-3′	131
Circ-Zfp236	Circ-Zfp236-F3: 5′- tccccgttcctacctggcca-3′ Circ-Zfp236-R3: 5′- cgggctcagacagttccaga-3′	140
mmu_circ_0000705	circ_0000705-F1: 5′-tcaagatgaagtcgttcccac-3′ circ_0000705-R1: 5′-acattctctctcggtgcttg-3′	143
mmu_circ_0000705	circ_0000705-F2: 5′-gaacatgtgcgcatggtggac-3′ circ_0000705-R2: 5′-gctgtcgtgggaacgacttc-3′	164
mmu_circ_0008590	circ_0008590-F1: 5′-caggggcaggatcagaacgc-3′ circ_0008590-R1: 5′-ctgtctcgttcgttcctccac-3′	160
mmu_circ_0008590	circ_0008590-F2: 5′-cgtccgccaagtcatcagat-3′ circ_0008590-R2: 5′-cttgtcggtgcgttctgatc-3′	141
mmu_circ_0012931	circ_0012931-F1: 5′-tccacttgttaagatacctc-3′ circ_0012931-R1: 5′-gcaagagtagatacataattcc-3′	168
mmu_circ_0012931	circ_0012931-F2: 5′-tatgaacatcatcacaggtc-3′ circ_0012931-R2: 5′-gcataactaatctgaggtatctta-3′	226
chr10:108583875-108691063	chr10:108583875-108691063-F1: 5′-tgggtggcttatctttccgc-3′ chr10:108583875-108691063-R1: 5′-gaaggtagtatactcacatggg-3′	211
chr10:108583875-108691063	chr10:108583875-108691063-F2: 5′-ttcatagcaagagaaactgg-3′ chr10:108583875-108691063-R2: 5′-ttggttcaagcggaaagata-3′	139
chr15:39566944-39616510	chr15:39566944-39616510-F1: 5′-actcagccaaaccgtgctat-3′ chr15:39566944-39616510-R1: 5′-ctagtagcttcatatgatcgac-3′	170
chr15:39566944-39616510	chr15:39566944-39616510-F2: 5′-tgctcactggagaagaatga-3′ chr15:39566944-39616510-R2: 5′-tctatatccatagcacggtt-3′	172
chr4:43091229-43115160	chr4:43091229-43115160-F1: 5′-ctgccgcccagtgtttaaat-3′ chr4:43091229-43115160-R1: 5′-gaccatgatggaatgtgtagac-3′	159
chr4:43091229-43115160	chr4:43091229-43115160-F2: 5′-actaaaatattcagtgtgtaactt-3′ chr4:43091229-43115160-R2: 5′-tatgtgttaaatttaaacactg-3′	175
β-actin	β-actin-F1: AGGGAAATCGTGCGTGACAT β-actin-R1:GAACCGCTCATTGCCGATAG	150
Cir- SIRT1-623	Cir- SIRT1-623-F3: GAGCAGGTTGCAGGAATCCA Cir- SIRT1-623-R3: ACAAAAGTATATGGACCTGA	136
Cir- SIRT1-395	Cir- SIRT1-395-F2: TTCAAGTTTGCAAAGGTCCA Cir- SIRT1-395-R2: AATCTGCCACAGTGTCATAT	137
Cir-CTGF-212	Cir-CTGF-212-F1: CTAGAGGAAAACATTAAGCCT Cir-CTGF-212-R2: ACAGGTCTTAGAACAGGCG	116
rno_circ_003172	rno_circ_003172-F2: GTCCACACTCCGGGATGAG rno_circ_003172-R2: AGCTCGTCCTTCACTGCGC	165
rno_circ_002671	rno_circ_002671-F1: CCACCAACAGATTCAGGAA rno_circ_002671-R1: CTCTTGAGTATCTGGTTCTG	129
rno_circ_002276	rno_circ_002276-F1: ACAAGAAGCTTGCTCAGGTC rno_circ_002276-R1: ATGTTCTGTGGCTCCTTGCT	163
rno_circ_001216	rno_circ_001216-F2: GGTGCCTCCAAGGAGGTG rno_circ_001216-R2: ACACACCGCCATGCAGTACTC	171
rno_circ_001215	rno_circ_001215-F2: GCGGTGCCTCCAAGGTTCC rno_circ_001215-R2: ACGGCCTTCTTGTCAGCTTTGG	217
rno_circ_000987	rno_circ_000987-F2: CTGGTGTCAAGTAAGGTATT rno_circ_000987-R2: TGAATAGAAGGGTACATCTG	181
rno_circ_NF1-419	rno_circ_NF1-419-F2: AGTCGAATTTCTACAAGCTTC rno_circ_ NF1-419-R3: AGCTTCTCCAAATATCCTCAT	179

**Figure 3:** **CircRNA NF1-419 influences the gut microbiota composition and cholinergic system.** (**A**) The circRNAs of *circ_zfyve1-504*, *circ_zcchc11-811*, *circ_zfp652-1147*, *circ_zfp236-1257*, *circNF1-419* and *circ_zranb1-1575* by reverse transcription polymerase chain reaction in *Ganoderma lucidum* extractions (LZ) (oral LZ of 50 mg/[kg·d]) and *Hericium erinaceus* extractions (HE) (oral HE of 50 mg/[kg·d]) treated SAMP8 mice brain samples lasting 24 weeks. (**B**) Over expression of *circNF1-419* in brain could change the gut microbiota at phylum (**a**) and genus level (**b**) of SAMP8 mice, see also in Supplementary Figure 8. (**C**) Expression of the proteins AChE, AMP, CHRNA1 and CHRNB1 in the brain tissues of SAMP8 mice after infection of over-expressing *circNF1-419* AAV. (**D**) Expression of the proteins AChE, AMP, CHRNA1 and CHRNB1 in the brain tissues of 12-month-old mice after infection of over-expressing *circNF1-419* AAV. (**E**) Expression of the proteins AChE, AMP, CHRNA1 and CHRNB1 in the brain tissues of 2-month-old mice after infection of over-expressing *circNF1-419* AAV. Data are presented as the means ± SD of more than 8 independent experiments, and more than 3 independent experiments in Western bolting. ^*^p <0.05 and ^**^p <0.01 *vs*. the model group by one-way ANOVA, followed by the Holm-Sidak test.

First, we utilized our previous designed AAV viral transduction system with RNA interference (*sicircNF1-419*) and separately an over-expressing *circNF1-419* (*sscircNF1-419*) (Supplementary Figure 4). Two microliters of the AAV packaging system (virus titer 1 × 10^12^) were injected into the cerebral cortex of SAMP8 mice. Statistical analysis of the 16S rRNA gene sequencing data showed that ss*circNF1-419* can significantly change the gut microbiota composition of the SAMP8 mice 7 weeks after infection – the relative abundance of Bacteroidetes, Actinobacteria, Deferribacteria and Cyanobacteria were increased (Figure 3B, *p* < 0.05 vs SAMP8 group) at the phylum level, and the relative abundance of *Bacteroides*, *Alloprevotella*, *Lactobacillus*, *Lachnoclostridium* and *Ruminiclostridium 9* were changed (Figure 3B, *p* < 0.05 vs SAMP8 group) at the genus level. Previous studies indicated that people who eat plenty of protein and animal fats have predominantly *Bacteroides* bacteria, while for those who consume more carbohydrates, *Prevotella* species dominate, which is due to the fact that the main sources of energy for *Bacteroides* species in the gut are complex host-derived and plant glycans [40]. Studies have revealed that the presence of *Prevotella* in the human gastrointestinal tract is inversely correlated with Parkinson’s disease [41, 42], and members of the family Lachnospiraceae could protect against colon cancer in humans by producing butyric acid with the functions of anti-inflammation and immunomodulation [43]. Histopathological observations showed that *circNF1-419* could improve the damage of intestinal tissues in SAMP8 mice and 12-month-old mice (Figure 4A), expression of AChE and AMP, CHRNB1 and CHRNA1 in the brain were improved (Figures 4C–4D), and expression of NF-κB p65 was activated (Figure 19B, *p* < 0.05). This all indicated that *circNF1-419* in the brain could improve the central cholinergic system and improve intestinal physiology in AD-like mice.

**Figure 4:** **CircNF1-419 changes the gut microbiota genetic trajectory in newborn KM mice.** (**A**) Intestinal physiology changes after infection of over-expressing *circNF1-419* AAV. (**B**) Heatmap of gut microbiota *in fimo* at phylum level after infection of over-expressing *circNF1-419* AAV in young mice. (**C**) Heatmap of gut microbiota *in* *fimo* at genus level after infection of over-expressing *circNF1-419* AAV in young mice. Data are presented as the means ± SD of more than 8 independent experiments. ^*^p <0.05 and ^**^p <0.01 *vs*. the model group by one-way ANOVA, followed by the Holm-Sidak test.

### *CircNF1-419* changes the gut microbiota genetic trajectory in newborn KM mice

To elucidate how *circNF1-419* in the brain influences the gut microbiota, we hypothesized that new discoveries could be found via monitoring the colonization of gut microbiota in newborn KM mice. Two microliters of the AAV (over-expressing *circNF1-419*) packaging system (virus titer 1 × 10^12^) were injected into the cerebral cortex of 2-week-old KM mice, whose mother was fed with standard diet or the HSHF diet.

Histopathological observations showed that *circNF1-419* could improve the damage of intestinal tissues in mice fed with the HSHF diet (Figure 4A). 16S rRNA gene sequencing revealed that the relative abundance of Bacteroidetes, Actinobacteria, Deferribacteria and Cyanobacteria were changed (*p* < 0.05 vs normal group, Figure 4B) at the phylum level, and the relative abundance of *Bacteroidales S24-7 group*, *Lachnospiraceae NK4A136 group*, *Alistipes*, *Alloprevotella*, *Lachnospiraceae*, *Bacteroides*, *Desulfovibrio*, *Lactobacillus*, *Roseburia* and *Helicobacter* were changed (*p* < 0.05 vs normal group, Figure 4C) at the genus level 8 weeks after infecting with the AAV. The expression of AChE and AMP, CHRNB1 and CHRNA1 were improved (Figure 3E, *p* < 0.05). Additional findings were that interference of *circNF1-419* aggravates some initial bacteria imbalance, including increasing the abundance of Actinobacteria, Deferribacteres, Proteobacteria while decreasing the Firmicutes (Figure 4B–4C), and *circNF1-419* could improve these changes. This indicated that the gut microbiota had notable correlation with the host, and this certainly included the circRNAs.

### Association analysis of *circNF1-419*, intestinal transcriptome and gut microbiota

To understand how *circNF1-419* influences the gut microbiota, we integrated analysis of the association between gut microbiota (Figure 3B and 4C) and differential expression mRNAs of the small intestine tissue (Supplementary Figure 5A–5B) on the *circNF1-419* treated SAMP8 and KM mice. As shown in Figure 3, *circNF1-419* in the brain mainly influences the bacteria *Candidatus Arthromitus*, *Lachnospiraceae FCS020 group*, *Lachnospiraceae UCG-006*, and [Eubacterium] *xylanophilum group*, and the mRNAs of *Gal3st1* (galactose-3- O-sulfotransferase 1), *Gamt* (guanidinoacetate methyltransferase), *Gpr62* (G protein-coupled receptor 62), and *Opalin* (oligodendrocytic myelin paranodal and inner loop protein). The relative abundance of those bacteria shown in Figures 3B and 4C, and the expression of mRNAs shown in Supplementary Figure 5A–5B, indicated that *circNF1-419* in the brain plays a role on multiple targets in the intestine, but how *circNF1-419* influences these mRNAs and the gut microbiota still needs considerable work on their metabolomics, signaling pathways and electrophysiology.

The mRNAs of brain tissue showed that the expression of GABRA1, GABRA6, St6galnac4, St8sia5, Pde9a, Tmem132a, Tmem163, Tmem62 and Tmem63c (Figure 5A and 5B) were up-regulated after over-expressed *circNF1-419* in brain, which indicated that the central immune system were activated, in other words that *circNF1-419* could activated central immune to improve the symptoms of AD, but need much more further study. And the Kyoto Encyclopedia of Genes and Genomes (KEGG) enrichment of 16S functional gene prediction analysis using PICRUSt also showing altered signaling pathways (Figure 5C) and the network (Figure 5D). Although the function and signaling pathway need much more studies.

**Figure 5:** **Association analysis of *circNF1-419*, intestinal transcriptome and gut microbiota.** Influences on the expression of GABRA1, GABRA6, St6galnac4, St8sia5, Pde9a (**A**), Tmem132a, Tmem163, Tmem62 and Tmem63c (**B**) in brain tissues. Kyoto Encyclopedia of Genes and Genomes (KEGG) enrichment of 16S functional gene prediction analysis using PICRUSt also showing altered signaling pathways (**C**) and the network (**D**). Data are presented as the means of more than 8 independent experiments, see also in Supplementary Figure 4.

### Circular RNA *circ_0001239* changes the gut microbiota genetic trajectory in mice

Additionally, we designed another AAV viral transduction system with RNA over-expressing mmu_*circ_0001239* (*ZCCHC11*, Supplementary Figure 6). The function of this circRNA in the brain was unknown but its expression was increased in the APP/PS1 and SAMP8 mice (Figure 4A). Two microliters of the AAV packaging system (virus titer 1 × 10^12^) were injected into the cerebral cortex of 7-day-old mice. After 3 months continuous infection, the gut microbiota composition was detected using 16S rRNA gene sequencing. The results revealed that *circ_0001239* can change the alpha diversity (Figure 6A) and beta diversity (Figure 6B) of the gut microbiota. The ternary phase diagram showed that the most of the bacteria were closed to the *circ_0001239* group (Figure 6C), and the relative abundance of different bacteria is shown in Figure 6D (*LDA* < 3.5), for example increases in the *Lachnospiraceae NK4B4* group, *Lachnospiraceae* and *Lactobacillus*, which indicated that over-expression of *circ_0001239* in the brain could change the genetic trajectory of the gut microbiota.

**Figure 6:** ***Circ0001239* changes the gut microbiota genetic trajectory in new born mice.** (**A**) The alpha diversity (**A**) and beta diversity (**B**) of the gut microbiota when the *circ0001239* over expressed in brain, see also in Supplementary Figure 6. (**C**) The ternary phase diagram showed that the most of the bacteria were closed to the *circ_0001239* group. (**D**) The relative abundance of different bacteria when the *circ0001239* over expressed in brain (*LDA* < 3.5). Data are presented as the means ± SD of 8 independent experiments. ^*^p <0.05 and ^**^p < 0.01 *vs*. the model group by one-way ANOVA, followed by the Holm-Sidak test.

The miRNA and mRNA sequences of brain tissues from the *circ_0001239*-treated mice showed that expression of mmu-miR-452-5p, let-7j and miR-205-5p were down-regulated (Figure 7A, |log2(FC)|≥1, FDR≤0.05) compared to the control, and there were 10 mRNAs up-regulated while seven were down-regulated (Figure 7B). Most previous studies on miR-452-5p [44, 45], let-7 [46, 47] and miR-205-5p [48, 49] focused on cancers. KEGG analysis of the mRNA sequences indicated that over-expression of *circ_0001239* in the brain mainly influences the ribosome and proteoglycans in cancer pathways, suggesting that *circ_0001239* has the sponge miRNA function and mediates a series of chain reactions in the brain, then influences gut function and microbiome engraftment from their parent.

**Figure 7:** **Effects of over expressing *circ_0001239* on KM mice brain.** (**A**) Nile red (red) and DAPI (blue) staining of BV2 cells bearing ss-ctrl or ss-circ0001239. Representative of three independent experiments. (**B**) MiRNA levels in over expressing *circ_0001239* KM mice brain samples. Representative of three independent experiments. (**C**) Differently expressed mRNA in over expressing *circ_0001239* KM mice brain samples. Representative of three independent experiments.

## CONCLUSIONS

This study revealed that the gut microbiome could influence the expression of some circRNAs in the brain, and reverse experiments indicated that over-expression of some circRNAs in the brain can influence the gut microbiota composition and their heredity to the descendant. As, over-expression of *circNF1-419* in the brain using an AAV viral transduction system, altered the gut microbiota structure and intestinal homeostasis. These results are the first demonstration of a link between circRNAs and the gut microbiome. They enlarge the ‘microbiome-transcriptome’ linkage library, providing more information on the interplay between gut and brain to aid in the identification of potential therapeutic markers and mechanistic solutions to complex problems commonly encountered in pathology, toxicology, and drug development studies. Additional studies will be required on these complex interaction systems.

## MATERIALS AND METHODS

### Animals

Male SAMP8 mice (5 months old, mean body weight 20 ± 5 g) were purchased from Beijing HFK Bioscience Co., LTD (Certificate No: SCXK [Jing] 2014-0004), and adult KM mice (18-22 g, 16 female and 8 male, 8 weeks old) were obtained from Center of Laboratory Animal of Guangdong Province, SCXK [Yue] 2008-0020, SYXK [Yue] 2008-0085). All the mice pair-housed in plastic cages in a temperature-controlled (25 ± 2°C) colony room with a 12/12-h light/dark cycle. The animals had free access to food and water. All experimental protocols were approved by the Center of Laboratory Animals of the Guangdong Institute of Microbiology. All efforts were made to minimize the number of animals used. All animals were allowed to acclimate for at least 1 week prior to the initiation of the experiments.

Then, SAMP8 mice were randomly allocated into 3 groups of 8 animals each: SAMP8 model group, ss*circNF1-419*-OV-AAV infected group, and si*circNF1-419*-OV-AAV infected group, two μl of the AAV packaging system (virus titer 1 × 10^12^) were injected into the cerebral cortex.

The female KM mice were randomly allocated into 2 groups of 8 animals each, one fed with high sugar & fat diet, and the other fed with standard diet. A month later, the female mice were randomly re-allocated into groups of 2 animals each and one male mice, keep feeding the original diet to the end of pregnancy, then all the mice fed with standard diet. After births one week, two μl of the AAV packaging system (virus titer 1 × 10^12^) were injected into the brain.

Balb/c mice were obtained from the Center of Laboratory Animals of Guangdong Province of China, (SCXK [Yue] 2008-0020, SYXK [Yue] 2008-0085), conventional breeding to 12 months old, two μl of the AAV packaging system (virus titer 1 × 10^12^) were injected into the cerebral cortex.

### Histopathology and immunostaining

The brain, colon tissues were removed and fixed in the 4% paraformaldehyde at pH 7.4 for further pathological observation. These tissue samples were made into paraffin sections after drawing materials, fixation, washing, dehydration, transparency, dipping in wax, and embedding. Obesity related parameters or other related pathologic changes were measured. The brains of animals were dissected. A total of four brains from each group were fixed in 4% paraformaldehyde solution and prepared as paraffin sections. Sections were stained with hematoxylin-eosin (H&E).

### Microbiome analysis

Fresh intestinal content samples were collected before the fasting of the rats for 12 hour and stored at -80 °C. Microbial DNA isolated from the samples, with total masses ranging from 1.2 to 20.0 ng, were stored at -20 °C. The microbial 16S rRNA genes were amplified using the forward primer 5′-ACTCCTACG GGAGGCAGCA-3′ and the reverse primer 5′-GGA CTACHVGGGTWTCTAAT-3′, and the rat forward primer 5′-CCTAYGGGRBGCASCAG-3′ and reverse primer 5′-GGACTACNNGGGTATCTAAT-3′. Each amplified product was concentrated via solid-phase reversible immobilization and quantified by electrophoresis using an Agilent 2100 Bioanalyzer (Agilent Technologies, Santa Clara, CA, USA). After NanoDrop quantification of DNA concentration, each sample was diluted to a concentration of 1×10^9^ molecules/μl in TE buffer and pooled. 20μl of the pooled mixture was sequenced on an Illumina MiSeq sequencing system (Illumina Inc, San Diego, CA, USA) according to the manufacturer’s instructions.

### Metabolomic analysis

After the water maze testing, the serum was acquired. 80 μL serum were added into 240 μL of cold mixture methanol with acetonitrile (2:1, v/v), and 10 μL internal tagging standard (L-2-chlorine-phenylalanine, 0.3 mg/mL, dissolved in methanol) were added, vortex after 2 min, then extracted using ultrasonic extraction method for 5 min. After 20 min standing at -20 °C, centrifuge for 10 min at low temperature (14000 prm, 4 °C), 200 μL of supernatant loaded into a sample bottle with lining tube for LC - MS analysis (Waters UPLC I-class system equipped with a binary solvent delivery manager and a sample manager, coupled with a Waters VION IMS Q-TOF Mass Spectrometer equipped with an electrospray interface (Waters Corporation, Milford, USA). LC Conditions: Column: Acquity BEH C18 column (100mm × 2.1mm i.d., 1.7μm; Waters, Milford, USA). Data analysis as described previously (Han, et al.).

### RNA isolation and sequencing

Total RNA was isolated using Qiazol and miRNeasy Kits, including additional DNase I digestion. Then remove the ribosomal RNA using Ribo-Zero^TM^ Magnetic Gold Kit, enzymatic degradation of linear RNA using Rnase R enzyme. Add fragmentation buffer to be fragments, synthesize the first chain of cDNA with six bases random hexamers, then the buffer, dNTPs, RNase H and DNA polymerase I to synthesize the second chain of cDNA. Purification uing QiaQuick PCR kit and elution using EB buffer after terminal repairing, processing bases A, add sequencing joint. For next generation sequencing, 0.5 μg ribosomal RNA-depleted RNA was fragmented and primed. The sequencing libraries were constructed using Illumina TruSeq RNA Sample Preparation Kits and were sequenced by Illumina HiSeq^TM^ 2500 flowcell.

The bioinformatics analysis of RNA annotation, functional classification, functional enrichment and cluster analyses were performed [47, 50, 51].

### Computational analysis of circRNAs

The reads were first mapped to the latest UCSC transcript set using Bowtie2 version 2.1.0 [52] and the gene expression level was estimated using RSEM v1.2.15 [53]. For lincRNA expression analysis, we used the transcripts set form Lncipedia (http://www.lncipedia.org). TMM (trimmed mean of M-values) was used to normalize the gene expression. Differentially expressed genes were identified using the edgeR program [54]. Genes showing altered expression with p < 0.05 and more than 1.5 folds changes were considered differentially expressed. The pathway and network analysis were performed using Ingenuity (IPA). IPA computes a score for each network according to the fit of the set of supplied focus genes. These scores indicate the likelihood of focus genes to belong to a network versus those obtained by chance. A score > 2 indicates a <= 99% confidence that a focus gene network was not generated by chance alone. The canonical pathways generated by IPA are the most significant for the uploaded data set. Fischer’s exact test with FDR option was used to calculate the significance of the canonical pathway.

For circRNA expression analysis, the reads were to mapped genome using the STAR [55] and DCC [56] was used to identify the cirRNA and to estimate the circRNA expression. TMM (trimmed mean of M-values) was used to normalize the gene expression. Differentially expressed genes were identified using the edgeR program. miRanda [57] was used to predict the miRNA target of the circRNA. R was used to generate the figure.

### CircRNA verification by quantitative real-time polymerase chain reaction (qRT-PCR)

To validate the reliability of high-throughput RNA sequencing and to explore the expression of circRNAs during aging, the expression levels of circRNAs were examined by qRT-PCR. With reference to Memczak’s method [58], two sets of primers for each circRNA were designed using Primer Express software version 5.0 (Table 1): an outward-facing set which was expected to amplify only the circRNA, and an opposite-directed set to amplify the linear form.

Total RNA was extracted (TRIzol^®^ Reagent, Life technologies), digested using RNase R, and purified. cDNA was synthesized using a Geneseed^®^ II First Strand cDNA Synthesis Kit (Geneseed, USA). Outward-facing primers were designed to amplify the fragment across the junction from cDNA, then the fragment was sequenced by Sangon Biological Engineering Company (Shanghai China). QRT-PCR was performed using Geneseed^®^ qPCR SYBR^®^ Green Master Mix (Geneseed, USA), and PCR-specific amplification was conducted with an ABI 7500 (Applied Biosystems, USA). The expression of circRNAs was defined based on the threshold cycle (Ct), and relative expression levels were calculated via the 2^-ΔΔCt^ method. GAPDH served as an internal standard control with all reactions performed in triplicate.

### Western bloting analysis

Global brain tissue was dissected from treated mice (purchased from the Beijing HFK Bioscience Co., LTD [Certificate No: SCXK (Jing) 2014-0004]) and proteins extracted with radioimmunoprecipitation assay (RIPA) lysis buffer (Thermo Scientific^TM^ T-PER^TM^ Tissue Protein Extraction Reagent, 78510). The proteins were separated by sodium dodecyl sulfate-polyacrylamide gel electrophoresis and transferred onto polyvinylidene fluoride membranes. After blocking with 5% nonfat dry milk in Tris-buffered saline (20 mM Tris-HCl, 500 mM NaCl, pH 7.4) with 0.2% Tween-20 (Aladdin, T104863), the membranes were probed with antibodies overnight at 4°C, followed by incubation with a horseradish peroxidase-conjugated goat anti-mouse (Servicebio, G2211-1-A) or goat anti-rabbit (Servicebio, G2210-2-A) IgG secondary antibody (1:2000). The antibodies were as follows; anti-Abeita A4, -APOE, -BACE1, -p53 (abcam, 66064), -p16 (Affinity, AF0228), -p21, -p-Tau-396, -TNF-α (abcam, 9739), -p-Tau-202, obtained from Affinity as well as GAPDH (CST, 2118L) and β-Actin (CST, 4970S). Band intensity was quantified using ImageJ software (NIH).

### Statistical analysis

All data are described as the means ± standard deviations (SD) of at least three independent experiments. The significant differences between treatments were analyzed by one-way analysis of variance (ANOVA) test at *p* < 0.05 using statistical package for the social sciences (SPSS, Abacus Concepts, Berkeley, CA, USA) and Prism 5 (GraphPad, San Diego, CA, USA) software.

### Ethics approval

The animal protocols used in this work were approved by the Institutional Animal Care and Use committee of the Center of Laboratory Animals of the Guangdong Institute of Microbiology.

### Study limitations

There are several strengths with this study, but there are also limitations. For example, the study lacks a rescue test with single bacteria, so we have not identified the one-on-one contact between circNF1-419 and single bacteria, and therefore could not find the signaling pathway or linking ligament. Using targeted strains in germ-free mice with multi-omics studies to reveal the interaction of circNF1-419 on the microbiome-gut-brain axis, or using knock-out circNF1-419 mice are needed in the future for positive validations.

## Supplementary Material

Supplementary Figures

Supplementary Table 1
